This article has been retracted.

# Adverse Influences of Nonstrabismic Amblyopia on Quality of Life of Teenagers in China

**DOI:** 10.1155/2022/2621991

**Published:** 2022-09-07

**Authors:** Yakun Wang, Hong Wang

**Affiliations:** Department of Ophthalmology, Clinical Medical College, Yangzhou University, Yangzhou 225000, China

## Abstract

The aim of this study was to explore the influences of nonstrabismic amblyopia on quality of life in adolescents. Health-related quality of life (HRQoL) scale, a multidimensional construct that indicates a fundamental health outcome, was used to measure physical and psychosocial functioning of the adolescents. Forty teenagers with nonstrabismic amblyopia and 40 control teenagers without nonstrabismic amblyopia were recruited between April 2019 and July 2021. The anthropometric measures, body image, physical activity outcome, and HRQoL scores including physical health, emotional functioning, social functioning, and school functioning were compared between the two groups. The results revealed that teenagers with nonstrabismic amblyopia had less weekly sedentary time (*P* < 0.001), weekly total steps (*P* < 0.001), and worse school functioning (*P* = 0.0211) than control teenagers. No significant difference was found in anthropometric measures and body image between the two groups (*P* > 0.05). This study implied the needs for teenagers with nonstrabismic amblyopia to enhance physical activities. Teachers and parents are encouraged to pay more attention to teenagers with nonstrabismic amblyopia to improve their school functioning.

## 1. Introduction

Amblyopia is a neurodevelopmental disorder, affecting up to 5% of the general population [1]. For patients with amblyopia, monocular vision or binocular vision is decreased because of poor visual stimulation in childhood [2]. After uncorrected refractive errors, amblyopia is the second most common cause of poor vision in children and young adults [2, 3]. The most common amblyogenic factors include strabismus and anisometropia. Strabismus is noticeable, while other types of amblyopia were not easily to be recognized by parents. Children may go undetected until they are beyond the critical period of treatment efficacy. Anisometropic amblyopia shows high prevalence in school-age children [4, 5]. Despite it, investigations on nonstrabismic amblyopia in quality of life were very limited. This may be due to that nonstrabismic amblyopia is deemed less serious than strabismus-associated amblyopia, which has obvious emotional and psychosocial consequences [6, 7]. Moreover, many amblyopia-related studies focus on the effects of amblyopia treatment [8, 9] but not the condition itself, and recurrence of amblyopia occurs in 25% to 50% of children after successful treatment, and binocular vision rarely returns to normal after repair [10].

To assess the physical and social functioning, well-being, and mental health of children and adolescents, health-related quality of life (HRQoL) has aroused much interest [11]. Certain key aspects of health are not assessed by clinical or traditional physiological measurements but can be detected by HRQoL measures. Quality of life was defined as “the individual” perception of their position in life in the context of the culture and value systems in which they live and in relation to their goals, expectations, standards, and concerns by World Health Organization [12]. HRQoL is multidimensional and includes various subdimensions of subjective experience, such as social interaction, psychological well-being, physical activity, and school performance, reflecting individual self-assessment, perception of enjoyment and well-being, and satisfaction with functioning, life, and general health [13, 14]. In recent years, the evidence of the effects of amblyopia on HRQoL has been measured [15]. Literatures point out that amblyopia indeed influences the individual together with family members [16], but the way in which amblyopia treatment has changed and some studies demonstrating that HRQoL implications of amblyopia are dated. Therefore, it is essential to reevaluate whether the influence of amblyopia on HRQoL has altered by changes in clinical practice. A previous study demonstrated that nonstrabismic amblyopia influences the quality of life of adults [17]. Currently, few studies have evaluated perspective quality of life in adolescents with nonstrabismic amblyopia.

Considering the importance of studying HRQoL, we performed a study to reveal the effects of nonstrabismic amblyopia on HRQoL in adolescents.

## 2. Methods

### 2.1. Participants

The study was conducted following the Declaration of Helsinki and was approved by the ethnical committee of Northern Jiangsu People's Hospital. Participants were recruited by department of ophthalmology in Northern Jiangsu People's Hospital. Written informed consent was gained from a parent or legal guardian before testing their child and after explanation of the nature and possible consequences of the study. Persons who visited the hospital underwent a complete eye examination including ocular motility test, slit lamp examination, refraction, cover-uncover test, and dilated retinal evaluation. The inclusion criteria were set as follows: (1) aged between 12 and 18 and (2) diagnosed with amblyopia [18]. The exclusion criteria were set as follows: (1) with strabismus [19], (2) with severe diseases that influence the daily life, and (3) unwilling to join in the study (for both teenager participants and their parents). Finally, 40 teenagers (male = 28 and female = 12) with nonstrabismic amblyopia were included, and 40 healthy teenagers (male = 23 and female = 17) without nonstrabismic amblyopia were recruited between April 2019 and July 2021.

### 2.2. HRQoL

The Pediatric Quality of Life Inventory (PedsQL) [20], recommended by Khairy et al. as a simple, easy, and reliable model for assessing HRQoL [21], was used in our study. The PedsQL questionnaire had 23 items in total and was divided into 4 domains regarding physical functioning (8 items) and psychosocial health (15 items). The latter one was further divided into social functioning (5 items), emotional functioning (5 items), and school functioning (5 items). Each item was reversely scored and linearly transformed, and higher scores indicate better HRQoL [20]. The transformation was set as follows: 0 = 100, 1 = 75, 2 = 50, 3 = 25, and 4 = 0. Children completed the PedsQL questionnaire by themselves after instructions from our research team. Children's self-reported HRQoL and their parents perceived children's HRQoL total scores were recorded.

### 2.3. Body Image Perception

Parents were invited to identify the most similar image with body of their children among various silhouettes to evaluate the parent's body image perception about their children [22]. There are two different silhouettes, actual figure and ideal figure, selected by the parents. Actual figure is the image that is believed to be the most similar with their children. Ideal figure is the image that is desired for their children. Overestimation of the body image means that actual figure is larger than ideal figure and vice versa. The profile series were divided based on the BMI categories determined by Cole's cut-off values: 1: underweight status, 2: normal weight status, 3: overweight status, and 4: obese status. Profiles 1 and 2 correspond to underweight; profiles 3, 4, and 5 correspond to normal weight; profiles 6 and 7 correspond to overweight; profiles 8 and 9 correspond to obesity.

### 2.4. Anthropometric Measuring

BMI was calculated as weight/height^2^, which was used to assess the weight status of each participant according to Cole cut-off values by sex and age [23]. The units for weight and height were kilogram and meter. The waist/height ratio (WHTR) was calculated to reveal the cardiovascular risk with the cut-off value set as 0.5 [24, 25].

### 2.5. Physical Activity Variables

Sedentary time was monitored using ActiGraph accelerometry monitors (Actigraph, USA) and was analyzed using the ActiLife 6.13.3 software (ActiGraph) [26]. Accelerometers were fixed with an elastic belt around the waist in the right side. Teenagers worn the accelerometers for a week and removed the accelerometers when bathing, swimming, and showering. The Evenson cut points were used to calculate the minutes spent in physical activity per day [27]. Adolescents aged 5–17 were recommended by World Health Organization to perform at least one hour of moderate-to-vigorous PA (MVPA) per day [28], which was measured in this study, and at least 3 valid days were needed for inclusion in analyses.

### 2.6. Statistical Analysis

Data are expressed as *N* (%) or mean ± SD. All analyses were carried out using SPSS, version 22 (SPSS Inc. Chicago, IL, USA). Chi-square test and unpaired t test were applied. The significance threshold was set as *P* ≤ 0.05.

## 3. Results

### 3.1. Comparison of the General Information between the Two Groups

General information including age, gender, and parents' education of teenagers in the healthy control and nonstrabismic amblyopia groups was collected. As revealed in Table 1, there is no significant difference among general information between the two groups (*P* > 0.05).

### 3.2. Comparison of the Anthropometric Measures between the Two Groups

Teenagers in the healthy control and nonstrabismic amblyopia groups had no significant differences in BMI and WHTR (*P* > 0.05, Table 2).

### 3.3. Comparison of the Body Image between the Two Groups

Teenagers in the healthy control and nonstrabismic amblyopia groups had no significant differences in body image (*P* > 0.05, Table 3).

### 3.4. Comparison of the Physical Activity Outcomes between the Two Groups

Teenagers in the healthy control and nonstrabismic amblyopia groups had no significant differences in daily MVPA (*P* > 0.05). However, the nonstrabismic amblyopia group showed longer weekly sedentary time and less weekly total steps than the control group (*P* < 0.001, Table 4).

### 3.5. Comparison of HRQoL of the Teenagers between the Two Groups

Teenagers in the healthy control and nonstrabismic amblyopia groups had no significant differences in scores of physical health, emotional functioning, and social functioning (*P* > 0.05). However, the nonstrabismic amblyopia group showed less school functioning scores than the control group (*P* = 0.0211, Table 5).

### 3.6. Comparison of HRQoL of the Parent Proxy-Reports between the Two Groups

As revealed in Table 6, there are no significant differences in physical health, emotional functioning, and social functioning of the parent proxy-reports between the two groups (*P* > 0.05). However, the nonstrabismic amblyopia group showed less school functioning scores than the control group (*P* = 0.0017).

## 4. Discussion

The subtypes of amblyopia (strabismic and nonstrabismic amblyopia) are not only disturbance of the development of the visual system at different points but also primarily different pathologic processes [29]. Some previous studies revealed the negative influence of strabismic amblyopia (or its treatment) on life of quality [30–32] while that of nonstrabismic amblyopia remains unknown. The study was designed to investigate the anthropometric measures, body image perception, physical activity outcomes, teenager-self reported, and parent-reported HRQoL from 40 teenagers with nonstrabismic amblyopia and 40 control teenagers. There were no significant differences between the general information including age, gender, and family education level of the teenagers in the two groups (*P* > 0.05). In addition, body image is a multifaceted mental representation of our bodies and their emotional experiences that is constantly updated. During adolescence, due to the constant physical and cognitive changes occurring, body image concerns occur frequently, thus increasing the evaluation and attention to the body and appearance. Sociocultural influences and social comparisons internalize the ideal of beauty, which leads to negative body image and dissatisfaction with appearance [33]. Therefore, adolescence is a time of significant physical and social change that can lead to negative body image. Perception of body image is associated with BMI and WHTR. However, reports about amblyopia and perception of body image are rare. Here, we found that the two groups also exhibited no significant differences in anthropometric measures including BMI and WHTR and perception of their parents on the body image (*P* > 0.05).

Amblyopia is associated with academic scores in mathematics, reading, social science, and science [34]. Consistent with previous literature, we found that adolescents with nonstrabismic amblyopia have worse school functioning than control peers (*P* = 0.0211), which might be associated with the vision loss in leaning period. Besides school functioning, physical health, emotional functioning, social functioning are also important for adolescents. It was reported that the nonamblyopia group had significantly better motor competence on the physical activity than either the corrected amblyopia group or the noncorrected amblyopia group [35]. Moreover, quite a number of amblyopia patients believe that amblyopia affects their study and work to a certain extent and generally affects their lifestyle [36]. Previous study also showed that children with strabismus had lower physical health scores, worse emotional functioning, and school functioning than those without strabismus, while no difference was found in these parameters between child with our without amblyopia [37]. However, the present study revealed the no significant difference in physical health scores and emotional functioning between adolescents with or without nonstrabismic amblyopia (*P* > 0.05).

Moderate physical activity has positive association with high HRQoL (measured by the total PedsQL score) in children [38, 39]. According to meta-analyses by Wafa et al., children with higher physical activity levels had a better HRQoL [40]. The positive association of physical activity and HRQoL was consistent regardless of age, gender, weight, and socioeconomic characteristics [41]. In our study, adolescents with nonstrabismic amblyopia have longer weekly sedentary time and less weekly total steps than control peers (*P* < 0.001). Considering that adolescents with nonstrabismic amblyopia also had lower school functioning in HRQoL (*P* = 0.0211), the positive association of physical activity and HRQoL in nonstrabismic amblyopia was identified.

Moreover, HRQoL perceptions between children or adolescents and their parents are likely to be different with increasing age because the child may have a more complicated and distinct understanding of the world instead of simply accepting opinions from parents. Thus, Tsiros et al. made suggestions to attach importance to the parent's perceived HRQoL [42]. Williams et al. found that, compared with children below 12 years old, there is less agreement between child-reported and parent's perceived HRQoL for children at the age of 12 years [43]. In our research, the comparison results of the perceived HRQoL for their children in the two groups were no different from the teenager-reported HRQoL (*P* > 0.05), which is similar to a previous study [39]. Our study revealed that both teenager-reported HRQoL and parent's perceived HRQoL revealed the worse school functioning in nonstrabismic amblyopia (*P* = 0.0017), while there are no differences in physical health, emotional functioning, and social functioning (*P* > 0.05).

There are also some limitations in our study. First, participants were recruited from a small geographical area. Further studies are needed to determine whether the identified HRQoL is present nationwide. Moreover, many of the effects of amblyopia and/or its treatment on HRQoL are experienced by the children; however, parents' opinions and perspectives on treatment may directly or indirectly influence children's beliefs.

## 5. Conclusion

After controlling for gender, age, and education of parents, there is a significant difference in physical activities and social functioning between adolescents with or without nonstrabismic amblyopia, which highlights the needs for teenagers with nonstrabismic amblyopia to increase physical activities for improving physical health. Teachers and parents should pay more attention to teenagers with nonstrabismic amblyopia to enhance their school functioning.

## Figures and Tables

**Table 1:** General information of the participants.

Parameters	Healthy control	Nonstrabismic amblyopia	*P* value
Age	15.89 ± 1.57	15.64 ± 1.13	0.5242
Gender			0.3524
Male	*n* = 23 (57.5%)	*n* = 28 (70%)	
Female	*n* = 17 (42.5%)	*n* = 12 (30%)	
Mother's education			0.8565
Low	*n* = 7 (17.5%)	*n* = 11 (27.5%)	
Medium	*n* = 17 (42.5%)	*n* = 20 (50%)	
High	*n* = 6 (40%)	*n* = 9 (22.5%)	
Father's education			0.4669
Low	*n* = 3 (7.5%)	*n* = 5 (12.5%)	
Medium	*n* = 21 (52.5%)	*n* = 22 (55%)	
High	*n* = 6 (40%)	*n* = 3 (7.5%)	

Data are expressed as *N* (%) or mean ± SD. Unpaired *t* test or chi-square test was conducted.

**Table 2:** Anthropometric measures of the participants.

Parameters	Healthy control	Nonstrabismic amblyopia	*P* value
BMI	19.21 ± 2.15	20.55 ± 2.36	0.1107
Normal weight	*n* = 37 (92.50%)	*n* = 35 (87.50%)	0.7449
Overweight	*n* = 1 (2.50%)	*n* = 2 (5.00%)	
Underweight	*n* = 2 (5.00%)	*n* = 3 (7.50%)	
Obese	*n* = 0 (0.00%)	*n* = 0 (0.00%)	
WHTR	0.47 ± 0.03	0.48 ± 0.03	0.1626
Non at risk	*n* = 39 (97.50%)	*n* = 38 (95.00%)	0.5562
At risk	*n* = 1 (2.50%)	*n* = 2 (5.00%)	

Data are expressed as *N* (%) or mean ± SD. Unpaired *t* test or chi-square test was conducted.

**Table 3:** Body image of the participants.

	Healthy control	Nonstrabismic amblyopia	*P* value
Under	*n* = 6 (15.00%)	*n* = 4 (10.00%)	0.7563
Correct	*n* = 31 (77.50%)	*n* = 32 (80.00%)	
Overestimation	*n* = 3 (7.50%)	*n* = 4 (10.00%)	

Data are expressed as *N* (%). Chi-square test was conducted.

**Table 4:** Physical activity outcome of the participants.

	Healthy control	Nonstrabismic amblyopia	*P* value
Daily MVPA			0.0979
Meet	*n* = 17 (38.3%)	*n* = 10 (38.3%)	
Not meet	*n* = 23 (61.7%)	*n* = 30 (61.7%)	
Weekly sedentary time	6322.44 ± 424.03	6885.43 ± 522.14	<0.001
Weekly total steps	54,178.23 ± 9627.18	52094.66 ± 9232.84	<0.001

Data are expressed as *N* (%) or mean ± SD. Unpaired *t* test or chi-square test was conducted.

**Table 5:** HRQoL of the participants.

	Healthy control	Nonstrabismic amblyopia	*P* value
Physical health	73.16 ± 13.64	72.89 ± 14.27	0.3066
Emotional functioning	72.21 ± 13.89	71.69 ± 13.21	0.0724
Social functioning	74.37 ± 12.12	72.33 ± 10.89	0.6123
School functioning	76.88 ± 14.03	73.14 ± 12.73	0.0211

Data are expressed as mean ± SD. Unpaired *t* test was conducted.

**Table 6:** HRQoL of the parent proxy-reports.

	Healthy control	Nonstrabismic amblyopia	*P* value
Physical health	82.52 ± 15.31	79.46 ± 10.95	0.9788
Emotional functioning	75.47 ± 12.48	73.85 ± 12.76	0.0901
Social functioning	76.58 ± 14.75	75.73 ± 12.64	0.1514
School functioning	84.12 ± 13.96	78.44 ± 12.93	0.0017

Data are expressed as mean ± SD. Unpaired *t* test was conducted.

## Data Availability

Data used or generated in this study are available from the corresponding author under reasonable request.

## References

[1] Carlton J., Karnon J., Czoski-Murray C., Smith K. J., Marr J. (2008). The clinical effectiveness and cost-effectiveness of screening programmes for amblyopia and strabismus in children up to the age of 4-5 years: a systematic review and economic evaluation. *Health Technology Assessment*.

[2] Kanonidou E. (2011). Amblyopia: a mini review of the literature. *International Ophthalmology*.

[3] Webber A. L. (2018). The functional impact of amblyopia. *Clinical & Experimental Optometry*.

[4] Gupta M., Rana S. K., Mittal S. K., Sinha R. N. (2016). Profile of amblyopia in school going (5-15 years) children at state level referral hospital in Uttarakhand. *Journal of Clinical and Diagnostic Research*.

[5] Ganekal S., Jhanji V., Liang Y., Dorairaj S. (2013). Prevalence and etiology of amblyopia in southern India: results from screening of school children aged 5-15 years. *Ophthalmic Epidemiology*.

[6] Hatt S. R., Leske D. A., Adams W. E., Kirgis P. A., Bradley E. A., Holmes J. M. (2008). Quality of life in intermittent exotropia: child and parent concerns. *Archives of Ophthalmology*.

[7] Hatt S. R., Leske D. A., Kirgis P. A., Bradley E. A., Holmes J. M. (2007). The effects of strabismus on quality of life in adults. *American Journal of Ophthalmology*.

[8] Carlton J. (2013). Identifying potential themes for the child amblyopia treatment questionnaire. *Optometry and Vision Science*.

[9] Koklanis K., Abel L. A., Aroni R. (2006). Psychosocial impact of amblyopia and its treatment: a multidisciplinary study. *Clinical & Experimental Ophthalmology*.

[10] Birch E. E. (2013). Amblyopia and binocular vision. *Progress in Retinal and Eye Research*.

[11] Solans M., Pane S., Estrada M. D. (2008). Health-related quality of life measurement in children and adolescents: a systematic review of generic and disease-specific instruments. *Value in Health*.

[12] Group, WH (1994). Development of the WHOQOL: rationale and current status. *International Journal of Mental Health*.

[13] Petracci E., Cavrini G. (2013). The effect of weight status, lifestyle, and body image perception on health-related quality of life in children: a quantile approach. *Quality of Life Research*.

[14] Zhang L., Fos P. J., Johnson W. D. (2008). Body mass index and health related quality of life in elementary school children: a pilot study. *Health and Quality of Life Outcomes*.

[15] Carlton J., Kaltenthaler E. (2011). Amblyopia and quality of life: a systematic review. *Eye (London, England)*.

[16] Tailor V., Bossi M., Greenwood J. A., Dahlmann-Noor A. (2016). Childhood amblyopia: current management and new trends. *British Medical Bulletin*.

[17] Kumaran S. E., Rakshit A., Hussaindeen J. R., Khadka J., Pesudovs K. (2021). Does non-strabismic amblyopia affect the quality of life of adults? Findings from a qualitative study. *Ophthalmic & Physiological Optics*.

[18] Kates M. M., Beal C. J. (2021). Amblyopia. *Jama*.

[19] Gunton K. B., Wasserman B. N., DeBenedictis C. (2015). Strabismus. *Primary care*.

[20] Varni J. W., Seid M., Rode C. A. (1999). The PedsQL: measurement model for the pediatric quality of life inventory. *Medical Care*.

[21] Khairy S. A., Eid S. R., el Hadidy L. M., Gebril O. H., Megawer A. S. (2016). The health-related quality of life in normal and obese children. *Egyptian Pediatric Association Gazette*.

[22] Collins M. E. (1991). Body figure perceptions and preferences among preadolescent children. *International Journal of Eating Disorders*.

[23] Cole T. J., Flegal K. M., Nicholls D., Jackson A. A. (2007). Body mass index cut offs to define thinness in children and adolescents: international survey. *BMJ*.

[24] Ashwell M., Hsieh S. D. (2005). Six reasons why the waist-to-height ratio is a rapid and effective global indicator for health risks of obesity and how its use could simplify the international public health message on obesity. *International Journal of Food Sciences and Nutrition*.

[25] McCarthy H. D., Ashwell M. (2006). A study of central fatness using waist-to-height ratios in UK children and adolescents over two decades supports the simple message – ‘keep your waist circumference to less than half your height’. *International Journal of Obesity*.

[26] Migueles J. H., Cadenas-Sanchez C., Ekelund U. (2017). Accelerometer data collection and processing criteria to assess physical activity and other outcomes: a systematic review and practical considerations. *Sports Medicine*.

[27] Evenson K. R., Catellier D. J., Gill K., Ondrak K. S., McMurray R. G. (2008). Calibration of two objective measures of physical activity for children. *Journal of Sports Sciences*.

[28] Bull F. C., al-Ansari S. S., Biddle S. (2020). World Health Organization 2020 guidelines on physical activity and sedentary behaviour. *British Journal of Sports Medicine*.

[29] Tong L. M. (1997). Unifying concepts in mechanism of amblyopia. *Medical Hypotheses*.

[30] Buffenn A. N. (2021). The impact of strabismus on psychosocial heath and quality of life: a systematic review. *Survey of Ophthalmology*.

[31] Gunton K. B. (2014). Impact of strabismus surgery on health-related quality of life in adults. *Current Opinion in Ophthalmology*.

[32] McBain H. B., Au C. K., Hancox J. (2014). The impact of strabismus on quality of life in adults with and without diplopia: a systematic review. *Survey of Ophthalmology*.

[33] Senín-Calderón C., Rodríguez-Testal J. F., Perona-Garcelán S., Perpiñá C. (2017). Body image and adolescence: a behavioral impairment model. *Psychiatry Research*.

[34] Shin H. S., Park S. C., Park C. M. (2009). Relationship between accommodative and vergence dysfunctions and academic achievement for primary school children. *Ophthalmic & Physiological Optics*.

[35] Sá C., Luz C., Pombo A., Rodrigues L. P., Cordovil R. (2021). Motor competence in children with and without ambliopia. *Perceptual and Motor Skills*.

[36] Packwood E. A., Cruz O. A., Rychwalski P. J., Keech R. V. (1999). The psychosocial effects of amblyopia study. *Journal of AAPOS*.

[37] Wen G., McKean-Cowdin R., Varma R. (2011). General health-related quality of life in preschool children with strabismus or amblyopia. *Ophthalmology*.

[38] Shoesmith A., Hall A., Hope K. (2020). Associations between in-school-hours physical activity and child health-related quality of life: a cross-sectional study in a sample of Australian primary school children. *Preventive Medical Reports*.

[39] Masini A., Gori D., Marini S. (2021). The determinants of health-related quality of life in a sample of primary school children: a cross-sectional analysis. *International Journal of Environmental Research and Public Health*.

[40] Wafa S. W., Hamzaid H., Talib R. A., Reilly J. J. (2014). Objectively measured habitual physical activity and sedentary behaviour in obese and non-obese Malaysian children. *Journal of Tropical Pediatrics*.

[41] Wu X. Y., Han L. H., Zhang J. H., Luo S., Hu J. W., Sun K. (2017). The influence of physical activity, sedentary behavior on health-related quality of life among the general population of children and adolescents: a systematic review. *PLoS One*.

[42] Tsiros M. D., Olds T., Buckley J. D. (2009). Health-related quality of life in obese children and adolescents. *International Journal of Obesity*.

[43] Williams J., Wake M., Hesketh K., Maher E., Waters E. (2005). Health-related quality of life of overweight and obese children. *JAMA*.

